# Application of Big Data Clustering and Visual Communication in Business Website Interface Design

This article has been retracted.

**DOI:** 10.1155/2022/8523763

**Published:** 2022-08-18

**Authors:** Xuan Qu

**Affiliations:** Shandong University (Weihai), Weihai 264200, China

## Abstract

The interface design of commercial websites is used in this paper to demonstrate the application of big data clustering and visual communication technologies. This paper presents the new requirements of user integration, emotion, and personalization by analyzing the broad influence of big data clustering technology and visual communication on the design concept and design method of commercial website interface design. Then, focusing on the information of visual graphic elements in web interface design and discussing how structures, images, words, emotions, and other elements can convey information more effectively through graphic means, the information in the web interface is creatively divided into two types: implicit and explicit. The database for the interface interaction system is built as part of this paper, which also uses fuzzy clustering to organize the data from the interface retrieval database and the hierarchical structure design method of process constraints to carry out interface information interaction and big data fusion processing. According to experiments, this algorithm's accuracy can reach 95.75%, which is about 11% higher than that of other approaches. This study can offer a workable design strategy for a business website's user interface.

## 1. Introduction

Commercial websites exhibit a thriving trend with the growth of e-business. Users' aesthetic skills have continuously improved as e-commerce has gradually taken over as the primary method of mass consumption. Although their fundamental shopping needs have been satisfied, they have raised the bar for the design of business websites [1]. The readability of web pages is significantly impacted by the aesthetic psychology of page layout style. Visitors will feel at ease and willing to accept a web page with a reasonable layout, which will inevitably improve the web page's visual appeal and encourage visitors to watch it [2]. Web interface design differs from general graphic design and has its own design traits based on the characteristics of web interfaces. The theme of “information transmission” should be consistently emphasized in web page design. The term “visual communication design” refers to any design that employs visual symbols to communicate any type of information. Visual design, as the name suggests, is the communication between the designer and the intended audience [3]. “Visual symbol” and “communication” are the two fundamental ideas in visual communication. Mass consumers are no longer content with simple online shopping consumption; they are paying more and more attention to the experience of online shopping [4]. This is due to the ongoing satisfaction of mass material needs and the ongoing improvement of the mass aesthetic level. The most user-friendly interface for commercial websites is the interface vision. E-business companies are focusing more and more on the value of visual design for brand building as a result of the constantly shifting market conditions and user needs.

Currently, the majority of the information provided by the web interface is visual. Accordingly, web interface design should adhere to the general rule of visual communication since it falls under the design type of visual communication [5]. This means that web interface design's primary visual components and design principles should be consistent with this rule. With the rapid advancement of information technology over the past few years, including the Internet, the Internet of Things, cloud computing, and triple play, the target of interaction design has shifted from small data, non-intelligent entities, and virtual bodies to the ecological environment of big data and vast wisdom. Users can only communicate with the system using the big data information display interface, and they must decode data to access it [6]. The design of the interface's user interface can enhance the big data environment's capacity for big data operation, management, and scheduling. People can acquire new knowledge and produce new value by using big data. Every alteration in people's behavior, location, and even physical physiological data has now become data that can be analyzed and recorded with the advent of mobile terminal devices like smartphones. Big data-related technology development is the foundation for the visual display interface of big data information [7]. Data gathering, analysis, and presentation are the three main steps in the processing of big data. The data presentation is the secret to a big data information visualization interface. The interface interaction design of big data creates the big data information base through GUI and man-machine interface and uses related database access and scheduling technologies to realize the information interaction of big data. The interface interaction design of big data realizes information management and data interaction through heterogeneous and hierarchical distributed interfaces.

The big data clustering algorithm and visual communication theory are applied in this paper to the interface design of commercial websites, leading to the following innovations: (1) In this paper, the database for the interface interaction system is constructed. Using the hierarchical structure design method with process constraints, interface information interaction and big data fusion processing are carried out, and the data from the interface retrieval database are clustered using the fuzzy clustering method [8]. To speed up the design process, a user-centered design process for the interface for big data information visualization is also recommended. The demand investigation process is divided into four steps: data analysis, planning and design, verification, and testing. The database that was designed for the interface interaction system has a good capacity for processing and scheduling big data information, and the data recall is good, according to the test results. (2) This essay examines the value of visual information communication in the creation of web interfaces from the viewpoints of theme, color, and text, putting special emphasis on the rational design of theme, color, text, and other information in the interface. It is based on the core ideas behind the design of user interfaces for commercial websites. A few practical design principles and methodologies are advanced by simultaneously analyzing the graphical representation of information in existing web interface design works. It presents a novel point of view on how business websites' user interfaces are designed.

## 2. Related Work

Web page design is a new design based on new media. At present, the research on commercial web interface design abroad has been at the forefront of this aspect, but the research on commercial web interface design in China has not been paid attention to, and the complete theory is still not perfect.

Schneider C et al. conducted an analogy analysis of text images, color matching, layout, etc. from the perspective of visual design through literature research, questionnaire survey, case analysis, and other methods and obtained the visual characteristics of different types of shopping websites. At the same time, the influence of user experience on the visual interface of shopping website is explored, and five design application strategies are proposed [9]. Bennett et al. believe that with the gradual increase of users' personalized needs, user interface design will continue to innovate and provide users with more novel, unique, and diversified customized experiences [10]. Mcnely uses design, psychology, communication, aesthetics, and other methods to analyze the artistic factors, combined with a website case from the perspective of art and technology, and gives a web design scheme [11]. From the perspective of users, Yang et al. analyzed the interaction and visual beauty of interface design and the optimization of visual communication design and discussed the design strategies and development directions required for the visual communication design of shopping websites [12]. Mendoza and Marasinghe analyzed the implementation process of website instances according to the design of web pages; and summarized the technical characteristics, general steps, and attention issues of implementation [13]. Silvia et al. pointed out that the role of graphic elements in web interface design is not only to beautify the visual experience; it has the functions of reducing the user's memory burden, guiding users to browse the web for information, enhancing recognition, and keeping the interface style consistent [14]. Lee pointed out that when a viewer clicks to open a web page, the first thing that attracts their attention is a layout consisting of elements of different colors, shapes, and sizes. In this way, the browser will change from a seeker with an attitude of acquiring information to an aesthetic subject with aesthetic expectations; and in the instant perception of the layout style of the web page, a complete separation from the content of the web page is completed [15]. In order to improve the information interaction and data processing capabilities of the interface, Wu proposed an interface interaction design method based on big data processing technology [16]. Na et al. took the visual design of the e-business website as the research object, analyzed the visual design elements of the e-business website, and explored the visual communication design strategy of the e-business web interface with the theme of visual information communication [17]. Wang et al. proposed a big data information processing and interface interaction design method based on semantic feature analysis, using cloud resource scheduling technology to develop and design the interface interactivity system to improve the comprehensive fusion ability of big data [18]. This method is prone to the problems of correlation offset and low fusion degree of information output in the management of interactive information.

This article analyses and thoroughly discusses the design and implementation of the algorithm and suggests an interface design strategy for commercial websites based on big data clustering and visual communication. It is based on a careful examination of earlier literature. The important role of visual information communication in web interface design is examined in this essay from the viewpoints of theme, color, and characters, with an emphasis on the interface's rational design of theme, color, and characters. It is based on the fundamental guidelines for designing the user interface of commercial websites. The database for the interface interaction system is being constructed concurrently. The hierarchical structure design method with process constraints is used for processing big data fusion and interface information interaction, and the fuzzy clustering method is used for information clustering of the interface retrieval database. It presents a novel point of view on the layout of business websites' user interfaces.

## 3. Methodology

### 3.1. Big Data Clustering Algorithm and Visual Communication Design

Big data is a data set composed of data with complex structure, huge quantity, and numerous types. Big data technology refers to the skill of using advanced scientific methods to mine and analyze all kinds of massive data and obtain the required resources as quickly as possible [19]. In the era of big data, the demand information of mobile terminal users can be deeply mined and collected through big data technology, including data statistics, analysis, processing, and presentation. The key to big data information visual display interface lies in data presentation. The main way of data presentation is data visualization. Data visualization is used to output the analysis results of big data in a readable and visible form, so as to facilitate users to obtain relevant information effectively [20]. Big data has four remarkable characteristics: (1) A huge amount of data. (2) Data diversity. (3) Require fast response speed. (4) Low-value density. There have been significant changes in people's needs and lifestyles as a result of the information explosion. The products for mobile terminals have changed quickly as a result of this change and now offer a variety of cutting-edge features. Big data has a very brief life cycle, and it is ingrained in users' everyday activities. The associated big data cannot be used after the user's instant activity has ended. Big data is only useful when it is linked to human activities, according to this argument [21]. The data visualization of the big data information display interface displays the big data information in the interface through the design elements such as menus, buttons, texts, icons, and pictures and realizes interaction with them in order to support users in accomplishing their objectives and tasks. These enormous databases, created by tracking users' consumption patterns and usage patterns, will ultimately provide useful information for the design, resulting in effective design guidance and enhancing the level, performance, and user experience of mobile terminal interface design. The interface interaction design of big data creates the big data information base through GUI and man-machine interface and uses related database access and scheduling technologies to realize the information interaction of big data. The interface interaction design of big data realizes information management and data interaction through heterogeneous and hierarchical distributed interfaces. The amount of data in big data visualization is too large, and it is impossible to show all the data to users without any processing. Therefore, it is necessary to analyze the data from the perspective of the target users, so as to ensure that the thinking and operation process of users are very clear when communicating with the display interface. The user experience level and requirement design are shown in Figure 1.

Web page design is to arrange reasonable visual information elements on the specified web page according to the theme, and the main basis is visual physiology and visual psychology. Interface design is also a kind of cultural creation behavior and its materialized form with high practical value. In the design of interface interaction, it is necessary to process big data information under the embedded Linux kernel control model and combine TCP/IP server to control the integrated transmission and reception of big data. Information visualization can be regarded as two mutual mapping processes of coding and decoding: coding is to map data into visual elements such as shapes, positions, colors, characters, and symbols. Decoding is the analysis of visual elements. The two characteristics of visualization coding are efficiency and accuracy. Efficiency means that a large amount of information can be obtained quickly, and accuracy means that initial real information can be obtained by decoding. In the big data environment, the ability of big data operation, management and scheduling can be improved through interface interaction design [22]. Compared with the traditional business model, e-business requires more efficient recognition of customers' visual feelings, that is, users' visual experience of the website interface. Therefore, when designing the website, it is necessary to fully locate the target customer base, which has achieved higher recognition. Send is conducive to the promotion of goods, improve and also recognized, thus greatly improving the overall economic benefits of enterprises. As a new mass information media, the web interface has the following characteristics as well as the general information media characteristics: (1) The economy of the subject. (2) Advanced means. (3) The universality of the object. (4) Abundance of content. (5) Diversity of forms. (6) Interactive operation. Big data information is jumbled and huge, so all initial information cannot be presented in the interface design. In order to better enable users to decode, it is necessary to be user-centered in the process of “coding”, that is, interface design.

A good user interface for a commercial website can accurately communicate information to visitors while also exceeding their expectations for visual appeal and achieving seamless functionality and visual effects integration. This is yet another unavoidable outcome of rising Internet penetration. If the content of visual information has charm and characteristics, it is the embodiment of visual communication itself and is expressed in the design of data interfaces in addition to in the form of visual information. The key to determine whether visual information is quickly and accurately transmitted to users is how to reflect these visual information contents in an effective way. The process of transmitting information involves first analyzing the raw data and turning it into information. Information is the interpretation of data, and data are the symbol for storing information. Before being used for communication, initial data must be arranged, processed, and transformed into meaningful information. In the design of e-business web interface, from the perspective of visual information transmission, color design plays a very important role, which can show the style of the website and establish the image of e-business website. In addition, due to the interactive characteristics of web information transmission, the publication of web information becomes a cycle of continuous updating. However, the release of web design works does not mean the end of the design. Web designers must regularly or irregularly adjust and modify the web pages according to the feedback information of users and the business objectives of each stage of the website and cooperate with the business strategies of the website in different periods.

### 3.2. Business Website Interface Design Strategy

First, this paper builds the general model of interface interaction design and designs the big data information processing algorithm. The information from the interface retrieval database is then clustered using the fuzzy clustering method, and under the direction of the Linux kernel source code, the program scheduling and cross-compilation of the interface are carried out in order to realize the development of interface interaction design. Visual information with the same high and low context as text is presented in the big data information visualization interface. As a result, before designing, users must be categorized. The information displayed and the visualization techniques vary depending on the user. Additionally, color is a crucial component of website design. It is the primary tool for influencing readers' visual psychology and drawing attention. We should think about how the computer color system works since web design is created by computers. Commercial websites should first select a standard color; next, the auxiliary color is chosen based on the standard color. Additionally, the interface currently primarily disseminates information, so the amount of text on the web page is still substantial. A user can interpret the information easily and conveniently with the best intuitive transmission form by avoiding the text, which can occasionally make the spread of information of pictures and colors unclear and lead to misunderstanding. The cross-compilation control method is used to track and design the information fusion in the interface interaction process when designing the interface interaction in the big data environment. First, the big data information fusion and data scheduling methods are used to process and schedule the information in the interface interaction process. Users gain new experiences thanks to the use and promotion of big data technology, but it also forces interface design concepts to gradually depart from their conventional “user-centered” appearances and delve deeply into their true meanings. It establishes a new concept for interface design from a broader perspective, including the interaction between products and the interaction between users and products. When conducting user research, the requirements put forward by users are relatively vague, and it is impossible to directly choose the appropriate data to express them. It is necessary to split the requirements put forward by customers in detail until the smallest dimension can be displayed by using data. Next, we need to select each group of data and select the data that can best show the customer's needs to show each user's needs. The design framework of the commercial website interface is shown in Figure 2.

The cross bus control method is used to schedule the big data bus transmission at the interface interaction output end, and the information from the interface interaction is read and compiled in the embedded database. The two-dimensional effect is employed in this paper to remove extraneous pseudo-physical decoration, and all interface elements, including buttons and icons, are kept to a minimum. Use basic shapes such as squares, circles, and rectangles. The increased public demand for more individualized information will be met by the interactivity of Web pages, which will also encourage user participation and help users realize some of their wishes, needs, goals, and abilities. The most fundamental requirement of the information society for information transmission is timeliness. Web pages accurately depict the immediacy of the contemporary information society thanks to their quick transmission speeds. The architecture of the interface system is distributed and multi-threaded. It processes big data information in the bottom layer, creates a knowledge rule base and a model database, integrates the initial data using the techniques of association rule scheduling and model database retrieval, and performs model analysis and cross-compilation control in accordance with the data processing outcomes. The initiative of visitors to receive information and participate in information feedback can be increased by effective interaction in web interface design. In addition, it helps to explain the transmission's actual impact and expected deviation in order to adjust the next communication's communication strategy in a timely manner and effectively convey information. Information can be conveyed using graphics as both the information's subject and its medium. It must interact with people, in whatever form it takes. Information integration and induction are particularly crucial during the data collection and processing processes. In order to increase users' trust in products, this integration of fragmented information can be accomplished through effective interface design, which includes comprehensive integration of information content, service, and experience.

According to an analysis of the overall framework for designing interface interactions, the bottom algorithm for interface interactions is created using big data information processing technology, and the time domain function of big data distribution for interface interactions is as follows:

(1) $$\begin{array}{c} {\dot{x}}_{j}^{i}=f_{j}^{i}\left(x_{j}^{i},u_{i},u_{j}\right). \end{array}$$

In the formula, *x*_*j*_^*i*^ represents the number of data points for interface interaction transmission at the *j*th sampling node, and *i* represents the dimension of the underlying database for interface interaction:

(2) $$\begin{array}{c} x_{j}^{i}\in R^{n}. \end{array}$$

In the *m*-dimensional phase space, the order of the interface interaction design is given as *n*, when the interface interaction hierarchical feature distribution satisfies

(3) $$\begin{array}{c} u_{i}\in R^{m}. \end{array}$$

Cross-compilation is adopted for information clustering, and the output clustering attribute feature distribution of big data clustering is obtained as follows:

(4) $$\begin{array}{c} x={\left[\ldots ,x_{i},x_{j}^{i},\ldots \right]}^{T}\in R^{n\times N}. \end{array}$$

According to the interclass dispersion of big data distribution, the fuzzy clustering center function of big data interaction is obtained as follows:

(5) $$\begin{array}{c} \dot{x}=f\left(x,u\right). \end{array}$$

The cluster vector set of fuzzy hierarchical output is

(6) $$\begin{array}{c} X=\left\{x_{1},x_{2},x_{3},\ldots ,x_{n}\right\}\subset R^{s}. \end{array}$$

The information entropy is introduced into the cabin environment color image evaluation to determine the factor weight. If there are *m* website color design samples and *n* semantic factors, the original evaluation index data matrix *R*=(*r*_*ij*_)_*m*×*n*_ is formed:

(7) $$\begin{array}{c} R={\left[\begin{array}{cccc} r_{11} & r_{12} & \ldots & r_{1n}\\ r_{21} & r_{22} & \ldots & r_{2n}\\ \ldots & \ldots & \ldots & \ldots \\ r_{m1} & r_{m2} & \ldots & r_{mn} \end{array}\right]}_{m\times n}. \end{array}$$

For a certain semantic factor *r*_*j*_, there is information entropy:

(8) $$\begin{array}{c} e_{j}=-\sum_{i=1}^{m}P_{ij}\cdot \;\ln\;P_{ij},\\ P_{ij}=\frac{r_{ij}}{\sum_{i=1}^{m}r_{ij}\left(i=1,2,3,\ldots ,m;j=1,2,3,\ldots ,n\right)}. \end{array}$$

Calculate the proportion *P*_*ij*_ of the index value of the *i*th cabin ambient color sample under the *j*th factor:

(9) $$\begin{array}{c} P_{ij}=\frac{r_{ij}}{\sum_{i=1}^{m}r_{ij}}. \end{array}$$

Calculate the entropy *e*_*j*_ of the *j*th factor:

(10) $$\begin{array}{c} e_{j}=-k\sum_{i=1}^{m}P_{ij}\cdot \;\ln\;P_{ij},\\ k=\frac{1}{\ln\;m}. \end{array}$$

The structural information *Q*_1_ of the image that fuses the image edge and noise level metrics defined in this paper is as follows:

(11) $$\begin{array}{c} Q_{1}=S_{1}S_{2}. \end{array}$$

Finally, the structural information metric of the whole image is to average the structural information metric of each subblock in the image.

The information that must be displayed on the display interface, along with any related display components, can be identified after data analysis. A thorough planning and design process is then required. The user's specific feelings during the decoding process are the main factors being taken into account at this point. In light of this, user-centered planning and design should be given more attention. This study integrates user psychological and behavioral characteristics, simplifies complex instructions, and pays close attention to the needs and aesthetic preferences of the target audience in order to produce an intuitive and efficient interactive operation. To enhance integration and robustness of interface interaction control, the interface interaction system of big data information processing can be installed on the basis of a Windows system, cross-compiled by a Linux embedded system, and the association rules are scheduled in a collaborative environment.

## 4. Result Analysis and Discussion

This paper aims at optimizing the visual design of the commercial website interface, highlighting the theme features of the commercial website, and improving the user experience when using the website. How to improve the texture of the whole website by optimizing the design strategy, and at the same time, let users have a good user experience, is the design idea that this design practice based on design optimization should pay attention to. In the design of e-business websites, based on user experience and visual factors, the text fonts in web design generally adopt 14px as the standard font, 16px as the subtitle font, 18px as the title font, and 12px is often used for an introductory text. Because the hardware carrier displayed in the designed visual interface is different from the hardware carrier used in the current design, it needs to be tested on the spot to ensure the concrete effect of field use; including whether the dynamic effect is up to expectations and whether the color difference is acceptable. The data in this chapter are analyzed by SPSSStatistics software, and the important color image factors are obtained from color image adjective variables by factor analysis. First, the correlation of variables is tested by calculating the correlation coefficient matrix, reflection image correlation matrix, Bartlett, and KMO test. The results are shown in Table 1.

Under the basic idea of putting users first, the number of screens in the interface should be kept at 2-3 at first, so that the visual focus of users can be kept on the product information. Second, the category of commodities is re-divided, and the main column navigation is arranged at the top of the interface, and the secondary column navigation is placed at the top left of the interface, which belongs to the visual center of gravity and respects the user's usage habits. In the design of e-business web interface, the contrast between the background color and the text color in the interface should be as obvious as possible. In this paper, pictures with complicated backgrounds should be avoided to highlight the main text information of the products. In this chapter, the collected data are averaged, and the experimental results of website color evaluation are shown in Figure 3.

Faced with many similar products, mobile terminal users' expectations for products include some psychological expectations and emotional experiences besides their basic functions. This kind of emotional experience can be roughly classified into the following categories: freedom of use, pleasure of creation, and the freshness of vision and familiarity of operation., which can be realized through the design of emotional interaction.  Figure 4 shows the gravel map of the factor. Where the abscissa represents the number of factors and the ordinate represents the characteristic value.

The first factor, which has the highest characteristic value and contributes the most to explaining the semantic adjective variables of the original color image, is seen in Figure 4. In the later period, the ability declined. The commodity display interface, a secondary page accessed through classification and searching functions, is an extension of commodity information. On the layout, the detailed information of the goods should be displayed, which is convenient for users to understand and screen the goods. On the premise of maintaining the unity of visual style, the extension of commodity classification, through the way of guiding users, diverts users from the home page through different demand objectives, and reaches this interface. The following two indexes, error and accuracy, are selected to experiment with this algorithm. The errors of different algorithms are shown in Figure 5. The accuracy of different algorithms is shown in Figure 6.

The noise of the interface is caused by redundant interference information, which will distract the user's attention, so that the user cannot concentrate on the elements that directly express the function and behavior of the product, which will bring cognitive pressure to the user and hinder the speed and accuracy of information transmission. Improper fonts, ambiguous icons, unnecessary decorations, etc. are all interface noises. From the aspect of interface vision, a simple interface style can simplify the interface elements and reduce the user's irritability and fatigue when filling in information. In terms of color, you can embellish the interface through the main color, so that users can know where they are on the website. In visual design, if the highest signal-to-noise ratio is maintained to show information, the usability of the interface can be enhanced. In other words, it is necessary to remove these minor or interfering design elements without affecting the function, so as to improve the signal-to-noise ratio. Image quality evaluation results are shown in Figure 7.

The design strategy of this paper mainly analyses the visual elements such as color, text, and graphics of the web page from the perspective of visual information transmission, according to the theme of website design, and better applies these visual elements to the e-business web interface design, leaving a good first impression on users. The scores of users' experience of commercial websites before and after optimization are shown in Table 2.

An excellent website design should make the navigation system easy, natural, and clear to use. We know that readers' way of reading web pages is free and jumping, so we should make sure that no matter where readers are on the website, they are free to jump to other pages they want. This requires us to have attached links on all pages, and it is best to go in with one click. Experiments in this chapter show that the highest accuracy of this algorithm can reach 95.75%, which is about 11% higher than other methods. In addition, the database of the interface interaction system designed in this paper has a good ability of big data information processing and scheduling, and the data recall is good. This research can provide a feasible design scheme for the interface design of commercial websites.

## 5. Conclusions

Visual elements like colors, words, and images are displayed in the interface when designing a commercial website. These elements give the interface its appearance and enhance its content. In this study, the big data fusion processing and interface information interaction are finished using the hierarchical structure design method with process constraints, and the interface retrieval database's information clustering is finished using the fuzzy clustering algorithm. This paper examines the significant role of visual information communication in web interface design from the perspectives of theme, color, and characters while combining with the fundamental principles of commercial website interface design. It emphasizes the rational design of the theme, color, characters, and other information in the interface. The experiment demonstrates that the interface interaction system's database has good big data processing and scheduling capabilities, and the data recall is good. This algorithm's accuracy can reach 95.75%, which is about 11% higher than that of other approaches. This study can offer a workable design plan for the user interface of commercial websites. In addition, it offers a fresh viewpoint on the interface design of business websites. Due to a lack of resources and knowledge, there are still some issues that need to be resolved even though this paper has made some advances in the theory and practise of commercial website interface design. The graphical information used in the interface design of commercial websites will be the subject of additional research in the following step.

## Figures and Tables

**Figure 1:** User experience level and requirement design.

**Figure 2:** Design framework of the commercial website interface.

**Figure 3:** Experimental results of website color evaluation.

**Figure 4:** Gravel diagram of factor.

**Figure 5:** Error comparison of different algorithms.

**Figure 6:** Accuracy comparison of different algorithms.

**Figure 7:** Image quality evaluation results.

**Table 1:** Bartlett and KMO test results.

Kaiser–Meyer–Olkin measurement of sampling adequacy		0.891
Bart's sphericity test	Approximate chi-square	5397.847
	df	4.5
	Sig.	0.00

**Table 2:** Use the user rating scale.

Index	Original website design	Post-optimization design
Interface fluency	7.14	8.92
Visual comfort	7.62	8.87
Favorability	6.95	9.14

## Data Availability

The data used to support the findings of this study are available from the corresponding author upon request.
